# Strategies of Bioceramics, Bioactive Glasses in Endodontics: Future Perspectives of Restorative Dentistry

This article has been retracted.

**DOI:** 10.1155/2022/2530156

**Published:** 2022-07-30

**Authors:** S. Chitra, Nibin K. Mathew, S. Jayalakshmi, S. Balakumar, S. Rajeshkumar, R. Ramya

**Affiliations:** ^1^Department of Prosthodontics, Saveetha Dental College & Hospitals, Saveetha Institute of Medical and Technical Sciences (SIMATS), Chennai 600 077, India; ^2^National Centre for Nanoscience and Nanotechnology, University of Madras, Guindy campus, Chennai 600 025, India; ^3^White Lab, Materials Research Centre, Saveetha Dental College & Hospitals, Saveetha Institute of Medical and Technical Sciences (SIMATS), Chennai 600 077, India; ^4^Department of Pharmacology, Saveetha Dental College & Hospitals, Saveetha Institute of Medical and Technical Sciences (SIMATS), Chennai 600 077, India; ^5^Department of Oral Biology, Saveetha Dental College & Hospitals, Saveetha Institute of Medical and Technical Sciences (SIMATS), Chennai 600 077, India

## Abstract

Prevalently, there is a primary strategy to cure caries using restorative materials notably bioceramics. Existing synthetic materials stimulate natural tooth structure with acceptable interfacial bonding and esthetic and biomechanical qualities with better durability. Several bioceramics have been introduced and investigated for their potentialities as restorative materials. Biomineralization of tooth initiates repair and regeneration of natural dental tissue and reinstating the integrity of periodontium. In the evolution of bioceramics in the aspects of different essential composition for dental application, recent technology and modern strategies revolutionize the restorative dentistry. Bioglass is one among the important bioceramics as a restorative material, and by regulating the properties of the material, it is possible to construct improved formulation towards restoration. This article reviews the current revolution of endodontics, existing restorative materials, and technologies to be achieve for engineering materials with the better design.

## 1. Introduction

Recently bioceramics-based restorative materials possess a great interest due to their sealing behavior with mineralization potentiality. Lot many materials are emerging day by day to fulfil the required criterion; in that direction, biodentin and Novamin are emerging materials owing to their mineralization potentialities [1]. Many researchers pointed out that a relative restorative material should accommodate the bioactive molecules along with inherent antimicrobial characteristic features, which efficiently deter microbial biofilm formation that indiscriminates the colonization [2]. Dentist expectation is on materials that are easy to use and inexpensive and give long-lasting cure; hence, research is underway to develop and analyze such kind of materials [3].

Modern sealing materials have evolved with great challenges (toxicity, mechanical strength, and integration). Tracing their historical background, over 170 years ago, silver amalgam- (silver and mercury) based materials have been used to seal the cavities [4]. Later on, tin has been included into the silver amalgam compound [5], but the drawback of this material was, tin-mercury intermetallic phase easily corroded, leading to breakdown of the fillings. Copper (Cu), introduced into amalgam to eliminate the intermetallic tin-mercury phases, became modern amalgam materials with silver-copper-tin alloy powders along with mercury [6]. These materials survived with both chemical onslaughts and mechanical stability in the oral environment for longer duration. Later, researchers found that release of mercury from the fillings, contaminated and owing to its toxic behavior, increases risk (carcinogenicity, damage to the tooth socket and alveolar bone) to the oral environment. Therefore, alternatives to silver amalgam were fused with gallium-indium-tin alloy at room temperature; with this, silver-copper-tin mixture was combined and formulated as paste [7]. These filling alloys were also prone to corrosion, and toxicological reactions of gallium became a challenge. After this era, resin-based composites progressed as endodontic filling around 1960s [8]. Modernized dental composites consist of paste with the mixture of dimethacrylate monomers along with cross-linking including silane-coatings and ceramic particulates, and this composite paste was used to seal cavities. These resin-based composites have strength similar to amalgam; however, polymerization shrinkage in the resin tooth interface proved to be a dramatic disadvantage of these materials [9]. To overcome such adversities, calcium phosphate-rich apatite with phosphoric acid components and porous organic/inorganic compounds were tried [10]. Consecutively, resin/silica-based porcelain bioactive materials are being attuned to improve the standard of restorative materials [11].

## 2. Milestones in Dentistry

Dentistry evolved and has grown systematically; initially three centuries before started the journey towards the development in dental medicine; many excellent inventions have been introduced and still climbing to progress. In the field of restorative dentistry, American Dental Association recognized endodontics specialty in the year 1963; this field takes credit for their contribution in dental emergencies as defined in “The Surgeon Dentist” [12]. Followed by this, Chinese had clear ideology in dental caries; they introduced arsenical compound (alloy materials) to treat pulp. In this connection, Pierre Fauchard is known as the father of modern dentistry; he introduced concepts of endodontics [13]. Qureshi et al. explained that in the next level Phillip Pfaff took it further into another dimension; he initiated pulp capping using gold/lead in the year 1756 [14]. Then in 1809, for the first time, root canal filling with gold foil was experimented by Edward Hudson; furthermore, the authors also explained in 1834 phenols for canal irrigation [15]. It was reported that the first endodontic instrument was developed by Edwin Maynard (1838), then the most expected gutta-percha recommended by Watt in the year 1857, followed by obturation demonstrated by Bowman (1867) [15]. In this direction, in modern dentistry, electric current was applied and tested for pulp capping by Black in the year 1867, who also suggested zinc oxychloride as a pulp capping material [15]. Then, radiographs were evolved and became essential part of endodontics; dental X-ray instruments were used for diagnostic purposes after 1919 [16]. On the other hand, in restorative research, the first ceramic (calcium hydroxide) was introduced in the year 1920 to treat infected root canals. After 1993, revolutionary bioceramics materials were evolved for apical sealing, repair, and restorative purposes [15]. Fully reclining dental chairs were publicized in the year 1958; similarly, in the 1990s, aesthetic techniques have been introduced for tooth whitening [17]. On the other hand, in the aspects of diagnostics, laser light, dual wavelength spectrophotometry, thermistor, thermocouple, infrared thermography, fibre optic transillumination, and digital imaging fibre optic transillumination have been sequentially evolved for the better identification of the problems [18]. In this modern era, laser in dentistry, computer aided designing and computer aided milling, and Dental Operating Microscope (DOM) are the supporting tools for better activation of therapies [18].

## 3. Root Canal and Associated Problems

Enamel is the strongest mineralized part of the human body; beneath that layer, a hard portion is dentin existing above the gingiva. Inside the root there is a soft tissue known as pulp, which contains nerves, blood vessels, and connective tissues. This pulp mainly supports the growth of the root canal of the tooth during the development of infants and contains a mass of connective tissue recognized as endodontium [19]. Root is embedded with the jawbone, the pulp provides the moisture and nourish the tooth, and the damage of this pulp is known as the root canal problem, which arise most of the times due to the infections/microbial exposures. The pulp and root canal possess an importance in tooth development; however, a fully developed tooth can possible to survive without pulp and relative cells, since surrounding cells provide the nourishment to the teeth. Root canal therapy mainly includes three steps cleaning the root canal, filling the root canal, and adding a crown/filling [20].

The primary cause of root canal problems such as severe decay, serious infection, cavities, and gum disease also leads to the damage of pulp and soft tissue inside the canal (Figure 1).

Bioceramics are the potential candidates for endodontic sealing, and this class of materials consists of mineral trioxide aggregate (MTA), ERRM (EndoSequence root repair material) Putty, ERRM Paste, Biodentine, and iRoot FS (preloaded paste in a syringe with material delivery tips for intracanal deliverance), iRoot SP, MTA Fillapex, and BC Sealer MTA Plus, gutta-percha, and Bioactive glass. As of now, MTA is the gold standard material for restoration; however, this can be replaced by bioactive glasses by improvising the properties towards mechanical stability and early setting time.

## 4. Restorative Materials and Relative Problems

Gutta percha (GP) is generally used as an obturation material for filling, along with this GP bioceramics composites, glass ionomer cement, or amalgam-based materials were utilized to induce the mechanical bonding between the tooth structure and the materials. Hence, bioceramics composites are the most expected material for restoration; besides, they exhibit adorable bonding between teeth and restorative components. The most common complications in the root canal treatments are microbial infections that may be percolated due to the following reasons which leads to root canal failure. (i) Multiple root canals at a time in the same tooth may lead to failure due improper cleaning. (ii) unpredicted or undetected crack in the root, improper sealing, and problem with the restorative materials may provide a way to pave microbes inside the canals [21]. (iii) Dietary habituates, accident wounds, acids by fermentation, and pathological infections may lead to damage in enamel, dentin followed by the (iv) root canal and pulp. To overcome these circumstances, some tooth pastes were used to cure the enamel/dentin remineralization (sensitivity) in the early stage; some of the restorative materials were in the function for root canal sealing and pulp treatment. Deep cavity due to sensitivity, traumatic injury, and microbial exposure may lead to necrosis in the pulp dentin. Hence, pulp capping is one of the important and essential techniques used in dental restorations to secure pulp from necrosis. In this case, initially, calcium hydroxide is used as a pulp capping material followed by many bioceramics.

Endodontic problem is biofilm-mediated disease; it is mostly associated with growth of microorganisms on the surface of canals. Potential pathogenic sealant component/new approaches are required for disinfection. Zaneva-Hristova and Borisova-Papancheva and Vishwanath and Rao [22, 23] stated that gutta-percha is one of the best restorative materials that was discovered by John Tradescant in the year 1656; then it was introduced to medical society by William Montgomerie in the year 1925 [22, 23]. Traditional gutta-percha is a famous root filling material; it can only act as a filler material but does not possess the capability to completely seal the canal. Owing to the improper sealing, microbes will travel inside the canal; therefore, it is essential to fix this problem with sealer material. Regular sealers have their own setting time and shrinkage behavior; those kinds of materials may or may not bond with the core gutta-percha, and that gap also encourages the microbial invade. Hence, bioceramics-based materials entered into an endodontic restorative industry to revolutionize the restoration society. Bioceramics such as hydroxyapatite, bioactive glasses, calcium phosphates, and their derivatives, alumina, and zirconia are being used as tissue and joint replacement materials in both orthopaedics and dentistry [24, 25]; owing to their biocompatible and osteoconductive properties as well as chemical and dimensional stability. Generally, commercially available bioceramics sealers are composed of calcium silicates such as dicalcium silicate, tricalcium silicate, colloidal silica, calcium hydroxide, and calcium phosphate monobasic. Zirconium, bismuth oxide, and boron can used as a radiopacifier to analyze filling proficiency. Bioceramics are ideal restorative materials; since they are not affected by blood contaminations, sensitivity or shrinkage is not a problem like other sealant materials [26, 27]. They are hydrophilic in nature and induce long-term sealing due to hydration reaction that influences the formation of calcium hydroxide followed by dissolution into calcium and hydroxyl ions.

## 5. Bioceramics in Dentistry

Bioceramics materials are the best choice as an alternative for pulp capping, perforation repair, pulpotomy, root canal filling, and obturation of immature teeth [28, 29], while, setting of bioceramics, pH of the surrounding environment is enhancing up to 12, owing to the hydration reaction (dissolution of ions from the material matrix), which rapidly inhibits the microbial growth. Almost 90% of endodontic treatments are succeeded based on the reports. Failures in endodontics are mostly related to persistence of various pathological infections; root filling materials with the conflicting tissue reactions were very minimal extent. However, sealing materials and relative technique exhibited divergent qualities in terms of sealing with varying clinical performances. Most of the reports enumerate the essentiality of superior biocompatible endodontic sealer, whereas the exact demand in sealant materials is early setting time and it possibly should exhibit improved antimicrobial properties against pathogens, since the major cause of problem was generated due to pathogens and sealing efficiency that is essential than the biocompatibility. Calcium hydroxide is one of the important bioceramics in endodontics, and it has been used in different forms. This material is less effective to inhibit some microbial species as well as bioactivity; alternatively, it exhibits potential biocompatibility owing to their solubility [30]. It was reported that it does not fulfil the required criteria to become an ideal sealer and concluded that detailed evaluation is required to elaborately analyze the materials' properties in endodontic sealing [31]. Similarly, released ions interreacted and precipitated as a mineral apatite that induces the osteoconductive potential of the material. Thus, there is need of mineralization as well as antimicrobial properties in the sealing materials. Hence, bioactive glass modification towards a sealing material can potentially sort out this existing problem (Table 1).

Amalgam-based resin composite entered into the dental society in the year1833 [3], after the entry of amalgam, Pierce introduced zinc phosphate cement (1879) and it is a majorly used material in dentistry; these materials are ruled in the 18^th^ century [40]; at the same time, clove oils and zinc oxide-clove cements are popularized in this period [41, 42]. Calcium phosphate is the gold standard material for medical applications [43].

In the 19^th^ century, also progressive materials were grown; in this connection, polycarboxylate was introduced by Smith (1968) [40]; similarly, Wilson initiated glass ionomer cement (GIC [1972]) [44] and then MTA introduced in the year 1993 and got FDA approval in a short span [45]. Biodentine is a bioactive and biocompatible material, which potentially overcomes the limitations of calcium hydroxide and MTA [43]. Followed by several bioceramics, bioglass entered into the era of dentistry in the year 2004; demanding bioglass was integrated in toothpaste (Sensodyne®) in the name of Novamin®, and the remineralization efficacy of this material was sequentially reported, and then forth bioglass was potentiality investigated in periodontics, endodontics, and remineralization applications (Figure 2) [46].

## 6. Merits of Bioceramics

Incredible biocompatibility of bioceramics in a physiological environment owing to their similarity with natural mineral apatite encourages these materials for biomedical applications (Figure 3). Osteoinductive, osteoconductive, and bioresorbable properties enrich the bone tissue regeneration [47, 48]. Chemical bonding with the microstructure of tooth and antimicrobial properties induces the improved hermetic seal with tooth structure that leads to relevant dental applications. MTA is one of the best sealants and majorly being used among bioceramics; it has good solubility, improved bioactivity, acceptable antimicrobial properties, and sealing ability. MTA revealed superior biocompatibility with mesenchymal stem cell proliferation without genotoxicity and cytotoxicity according to earlier reports [49, 50]. Elevated solubility of MTA may jeopardise in long-lasting sealability in restorations, and it is critical to withstand like a bioactive material [51, 52]. Further, in this time period, biodentine was evolved; this is also formulated in a manner similar to MTA-based compositions with some improved properties. In the case of biodentine and MTA, calcium carbonate (CaCO_3_) acts a nucleation point to form the calcium silicate hydrate gel (C-S-H). Along with this material, water-soluble polymers balance the viscosity and induce the setting time. The setting time of biodentine starts at 6 minutes, and final setting occurs in about 45 minutes. This is one of the attractive behaviors of biodentine over other calcium silicate-based materials. Biodentine explicates improved mechanical stability and faster setting that lowers the risk of microbial/bacterial contamination than MTA [53]. EndoSequence Root Repair Material exhibited leakage in sealing compared to MTA groups. However, this material revealed similar antimicrobial and biocompatible properties related to MTA [54–56].

## 7. Uses of Bioceramics

The following are the uses of bioceramics:

1. Endodontics: obturation, sealers, retrograde filling, perforation repair, apexification, pulpotomy, and regenerative endodontics [27]
2. Restoration: dentin hypersensitivity, dentin substitute, dentin remineralization, and pulp capping [57]
3. Prosthetics: prosthesis, prosthetic device implants, implant coatings to improve osteointegration, and biocompatibility [58]
4. Surgery: fillings in surgical bone defects, joint replacements, alveolar bone augmentation, orbital floor fracture, and sinus obliteration [59, 60]

Bioceramics are prevalently used by the dental community; in this connection, MTA is a benchmark material in endodontics as well as restorative dentistry among bioceramics. However, some limitations are reported by several authors [27, 61]. Hence, based on the understanding from literary reports, it can be expected that up-to-date informative knowledge of new bioactive materials is essential to confirm the suitable materials based on the relevant clinical needs. [27] Modifying the glass network may produce new crystal lattices with required properties in bioactive materials that may enlighten the dentistry with the fulfilment of relevant desires. Biomaterials were drastically designed and developed towards dental research innovations in the last 9 years. Zirconia and relative bioactive scaffolds analyzed for bone regeneration and bioactive molecule demands were also identified in the last decade. Similarly, the importance of silver amalgam, alloys, and nonresinous cements was significantly decreased. Extensive focus is on restorative materials with enhanced regenerative potentiality, aesthetic restorative materials, and dental implants [62].

Bioactive components (Si, C, P, and Na) in restoration compositions induce the formation of mineral apatite crystals that leads to bonding integration in demineralized dentin, which is directly proportional to the incubation time in oral environment. Saliva itself has some essential ions along with that those relevant bioactive ions penetrate deep into dentin to regenerate dentinal tubules and also generate an entanglement that enhances the adhesive strength. Mineral apatite precipitation on the restorative materials produces beneficial interfaces on the adhesive restorations that encourages the remineralization and induce enzymatic reaction of collagen mesh followed by fossilization of metalloproteins [63]. It was reported that compared to current restorative materials, inclusion of bioactive glasses, tricalcium phosphate, and hydroxyapatite with the restorative composition positively triggers the chemical as well as biological properties [64, 65]. These bioceramics explicated tremendous biological, bioactive, and exceptional biocompatible properties. However, poor mechanical properties hinder their growth in dental application [66]. Hence, changes in the materials engineering possibly help to overcome this drawback in terms of incorporating mechanically stable ions in the lattices of host materials to reconstruct the crystallinity, material stability, and solubility that may provide a way for these materials into clinical dentistry [66, 67]. Implant failure can be overcome by coating bioactive materials on the implant surfaces in terms of inducing osteointegration, corrosion resistance, antimicrobial properties, and bone bonding ability, and coatings also enhance the biological fixation between metallic implant and bone [68, 69]. Implant biocompatibility and longevity also have positive stimulation on the regeneration of bone in the oral circumstances. It was also reported that direct coatings of therapeutic agents such as proteins, ligands, and growth factors provide beneficial osteoconductive properties, combat infection, stimulate bone growth, and also enhance the lifespan of implants [70, 71]. On the other hand, bioactive ceramics is being used as a coating material, since several metal implants and screws that are been used for dental treatments damage the tissue and interrupt the blood supply; therefore, cells die, inflammation occurs, and the interfacial atmosphere may be destroyed. Mostly, metals are used as dental materials; thus, there may be a chance of corrosion on the implant surface and corroded ions may percolate inside the tissues and cells that initiate the variety of clinical problems. These problems can be controlled by coating bioactive components on the porous metal surfaces [72].

## 8. Bioglass Journey in Dentistry

Dental resin bonding with tooth is a challenging criterion to overcome, due to the interaction between the hydrophobic resin and the hydrophilic surface of the tooth; despite this, it can be resolved by making resin composites with hydrophilic bioactive glasses (Table 2, Figure 4). Recently, researchers analyzed commercial polymer-based materials (AH plus and poly-c) to formulate a paste of bioglass, from which one of the major issues of bioactive glass with poly-c is the formation of crack, due to shrinkage at the time of drying and evaporation of liquid. Subsequent evaporation probably moves through the interrelated pores of the bioglass network towards inside of the surface, which might generate capillary stresses causing crack propagation. Comparatively, these stresses are smaller in powders than monoliths due to the evaporation path, which are capable of inducing fracture. Narrow porosity distribution with increased grain size can render this problem [73]. Shrinkage of sealant paste (bioglass and poly-C) creates a gap, which leads to poor mechanical properties and instigate failure of dental restorations. Some of the earlier reports towards the development of sealant are tabulated in Table 2.

Amandeep et al. [83] reported the detailed survey of some restorative materials such as zinc oxide eugenol, calcium hydroxide sealers, and resin-based sealers. Zinc oxide eugenol has long successive history over 100 years; however, prolonged setting time, solubility, and shrinkage are the major complications. Antimicrobial activities of calcium hydroxide sealers are appreciable, but solubility is the major disadvantage. Resin-based sealers have been successful over the past few decades due to its improved flowability; however, reduced adhesive property is yet to be overcome. Similarly, Patel et al. [84] reviewed the oroactive dental biomaterials for endodontic therapy and mentioned some limitations of biomaterials including polymers, metals, bioceramics, composites, and natural minerals. Structural stability, cytocompatibility, and mechanical resistance of polymers are not up to the requirement. A metal exhibits complexity in corrosion and challenges due to interaction with the physiological environment. In case of bioceramics, fabrication and processing are difficult; lower impact resistance and brittleness are the major issues. Composites exhibit foreign body reaction at physiological environment; correspondingly, rapid immunological problems were noted in natural materials. It has been reported that bioglass was able to maintain its stability more than two months while soaked in brain heart infusion media and also enumerated similar mechanical behavior rather than decreased fracture resistance compared to commercial materials. Hence, it is easy to construct the structure of bioactive glasses with the relevant properties than some commercially available endodontic sealants.

Generally, bioglass particulates are mixed with phosphoric acid to form a paste, which positively interacts with enamel surfaces and protects orthodontic brackets from erosive solution, as reported by Abbassy et al. [85]. Similarly, Ahmed et al. [86] elaborated that bioglass paste with diluted phosphoric acid has significant effect on remineralization of enamel lesion. Bioglass with 30% phosphoric acid is used to treat dentin hypersensitivity, and sealing was observed in depth of dentinal tubules by Lee et al. [87]. Bioglass formulation was available in commercial toothpaste, which remineralizes the eruption of tubules at the dentin/enamel. Continuous brushing by the respective toothpaste initiates tubule occlusion, by the development of apatite on their surfaces and fixed restorations on the margins to fill gaps, and can also eliminate secondary caries over a period of time [88]. In another report, Adanir et al. [89] studied the sealing ability of resin-based commercial root canal sealers such as Diaket, EndoREZ, and AH26 along with those of zinc oxide-eugenol-based U/P sealer and concluded that none of these sealers completely prevent the leakage of fluids, among which zinc-oxide eugenol exhibited more significant leakage. However, cytotoxicity is one of the major problems in most of the commercially available endodontic sealant materials [90, 91]. Milly et al. [92] evaluated that bioglass/polyacrylic acid treatment enhanced remineralization of enamel white spot lesion. Bioglass with polyacrylic paste was able to increase the surface area, mechanical properties, and mineral content, resulting in augmented mineralization [91].

Generally, bioceramics are the materials that exhibit mineralization, which simulate the natural mineral component on the canal voids of the tooth. Bioactive ions are released from the ceramics material in the exposure of oral fluid in that environment; mineral apatite tends to form over the restorative materials, which enhances the durability of the restoration. On the other hand, in the absence of bioactive ions, leached ions may not be having the potentiality to regenerate therefore it drops its stability. Bioceramics has the tendency to easily bond with polymer, and it became hardened; hence, it is accessible to use owing to its early setting time and stronger bonding nature. These positive features of bioceramics revolutionize the restorative society [20, 24]. Bioceramics are the most expected materials for restorative purposes; linear development in the aspects of composition was evolved with respect to duration. Initially, bioceramics journey started with calcium and phosphate compositions based on the silica, sodium, fluoride, zinc, carbon, iron, aluminium, bismuth, tantalum, ytterbium, barium, chlorine, sulfur, nickel, tungsten, titanium, silver, copper, tin, and mercury which have been included in different formulations depending on the need while growing ceramic materials. Currently, bioglass is the active material with different formulation and network chemistry. Hence, engineering glass network chemistry initiates the tunable characteristics such as porosity, morphology, structural aspects, degradability, bioactivity, and biocompatibility properties of the material. Besides, deep investigation and understanding the properties of bioglass lead to generate better restorative materials with acceptable stability as well as mineralization potentiality.

## 9. Summary and Future Direction

Starting from calcium silicate, so far, plenty of materials as well as many investigations have been reported in the aspects of various biocompatible and structural properties of existing ceramics. As of now, MTA (calcium silicate based bioceramics) is considered a potential candidate for endodontic restorative material owing to their biological characteristic feature and physicochemical properties. Followed by MTA, recently, biodentine is also gaining impactful attention due to their physico-bio-chemical properties; however, even more *in vitro* and *in vivo* studies are required to exactly assess the properties of this material. Addition of protein (CPNE7) into bioceramics may induce reparative dentin formations while using in pulp capping. Biodentine is similar in composition to that of bioglass, and not many reports are available to elaborate bioactive glass role in dentistry and also with the extended understanding in the characteristic features of the material at oral environment. However, based on the basic properties of bioglass, it can be assumed that it is one of the best materials for bioactivity among all bioceramics; however, this material has limitations in mechanical stability. By engineering stable bioglass with substituting strong metal ion in the glass network in terms of stronger metal ion in the lattice of bioglass or fabricating bioglass with hard polymer composite, it is possible to achieve better material for restoration. It is essential to analyze in detail, such kind of materials in the direction of structural, mechanical properties, and *in vitro/in vivo* compatibility.

## Figures and Tables

**Figure 1:** The most common stages of tooth problems.

**Figure 2:** Timeline for the evolution of restorative dentistry.

**Figure 3:** Schema explains the formulations of commercial restorative materials.

**Figure 4:** Bioactive material's impactful role in dentistry.

**Table 1:** The most common restorative materials with their compositions.

Name	Composition	References
Activa BioActive restorative	Powder: silicate bioactive glass, sodium fluoride silicate bioactive glasses, and sodium fluoride Liquid: diurethane modified hydrogenated polybutadiene, methacrylate monomers, altered polyacrylic acid, and distilled water	[32]
Cention N	Powder: barium aluminosilicate glass, isofiller, ytterbium trifluoride, calcium fluorosilicate glass, and calcium barium aluminum fluorosilicate Liquid: urethane dimethacrylate, tetramethyl xylylene diurethane dimethacrylate, tricyclodecane dimethanol dimethacrylate, polyethylene glycol 400 dimethacrylate, Ivocerin, and hydroxyperoxide	[33]
Mineral trioxide aggregate (MTA)	Mineral trioxide aggregate is a mixture of tricalcium silicate, dicalcium silicate, tetracalcium aluminoferrite, tricalcium aluminate, gypsum, and bismuth oxide. It is currently marketed mainly in two forms: GMTA (gray) and WMTA (white)	[34]
ERRM Putty, ERRM Paste (ERRM-EndoSequence root repair material)	Both ERRM putty and paste materials are composed of calcium silicates, calcium phosphate monobasic, tantalum oxide, and zirconium oxide	[35]
Biodentine	Biodentine comprises tricalcium silicate, zirconium oxide, calcium carbonate, and liquid-containing calcium chloride as a setting accelerator.	[34]
BC sealer and iRoot SP	Zirconium oxide, dicalcium silicate, tricalcium silicate, calcium silicates, colloidal silica, calcium hydroxide, and calcium phosphate monobasic	[34]
Endo CPM sealer Egeo	Calcium carbonate, silicon dioxide, bismuth trioxide, barium sulfate, sodium citrate, calcium chloride, and propylene glycol alginate	[36]
ProRoot Endo Sealer	Calcium sulphate, dicalcium silicate, tricalcium silicate, bismuth oxide, and traces of tricalcium aluminate along with water-soluble polymer viscous solution	[37]
AH Plus	Calcium tungstate, zirconium oxide, bismuth nitrate, epoxy resin, and silica	[38]
Sealapex	Calcium hydroxide, zinc oxide, barium sulfate, titanium dioxide, and zinc stearate	[38]
Zinc oxide-eugenol-based sealers	Zinc oxide, zinc acetate, rosin, and eugenol	[39]
Glass ionomer	Calcium aluminosilicate and polyacrylic acid	[39]
Amalgam	Silver, copper, zinc, tin, and mercury	[39]

**Table 2:** Importance of bioglass in the journey of dentistry.

Reports	Applications	Summarization	References
Deng et al. investigated the effect of 45S5 bioglass on bleaching efficacy of bovine enamel	Bleaching and whitening	Combination of bioglass and hydrogen peroxide could be a promising adjunct for bleaching therapy	[74]
Resin-modified glass ionomer cement bonded with dentin pretreated by bioglass using a variety of air abrasion techniques to evaluate the material and dentin bonding interfaces	Bonding durability and healing	Bioglass treated dentin samples explored better bonding with resin-ionomer cement and summarized that bioglass-treated surface exhibited improved remineralization and healing ability	[75]
Hydrated calcium silicate filler effect on resin-based pit and fissure sealant to prevent secondary caries, this was reported by Yang et al.	Caries prevention	Incorporation of calcium silicate in the pit resulted in changing the environment from a cariogenic state to a remineralization state	[76]
Gihan et al. explored the epoxy resin bioactivity and bond strength, after the incorporation of bioglass nanoparticulates	Endodontic sealer	Incorporation of 10% bioglass into epoxy resin is an effective method to encourage bioactivity without affecting bond strength	[77]
Evaluation of ionic dissolution and apatite forming potential of bioactive glass containing polydimethylsiloxane- (PDMS-) based sealant by Niko-Pekka et al.	Endodontic sealer	Bioglass containing PDMS caused higher absorption and ionic solubility than control; bioglass-PDMS revealed rapid mineralization and feasible antimicrobial properties	[78]
Mohn et al. analyzed the bismuth oxide and barium sulphate including bioactive glass particulates with high alkaline capacity and radioopaque properties for potential root canal dressing material	Root canal filling or dressing material	Bismuth oxide modified bioglass increases radiopacity, and alkaline behaviour promotes the sealing ability	[79]
Another study by Mohn et al. explained that polycaprolactone (PCL) or polyisoprene (PI) mixed 45S5 bioglass could create apatite interface, which ultimately acts as an endodontic sealer	Endodontic sealer	Bioglass filled PI and PCL composite materials resulting in improved bioactivity and immediate sealing	[80]
A study by Sfalcin et al. experimented that chemophysical properties of resin infiltrant (ERI) doped bioglass reduce water absorption and solubility	Treatment of white spot lesions	Resin infiltrant-bioglass enhances chemomechanical properties, such that innovative materials might prevent demineralization and induce remineralization on enamel surfaces	[81]
Wang et al. investigated the effect of Ca_3_SiO_5_/CaCl_2_ composite paste on setting time, compressive strength, bioactivity, and biocompatibility to explore the use in root canal filling	Root canal filling	Ca_3_SiO_5_/CaCl_2_ composite cement revealed biocompatibility and good bioactivity, a potential candidate as a root canal sealing material	[82]

## Data Availability

The data used to support the findings of this study are included within the article.
